The article "Study on the Relationship between Unexplained Recurrent Abortion and HLA-DQ Gene Polymorphism" was retracted in 2023. Reasons: signs of a paper mill; suspected computer-generated content; unreliable results or conclusions; lack of ethics approval or compliance.

# Study on the Relationship between Unexplained Recurrent Abortion and HLA-DQ Gene Polymorphism

**DOI:** 10.1155/2022/8005538

**Published:** 2022-08-29

**Authors:** Jie Tang, Jichao Zhu, Longwen Shu, Xiaohong Huang, Siming Ma

**Affiliations:** ^1^Department of Obstetrics and Gynecology, Huzhou Central Hospital, Huzhou 313000, China; ^2^Department of Laboratory Medicine, Huzhou Central Hospital, Huzhou 313000, China

## Abstract

**Objective:**

The study aimed to investigate the relationship between human leukocyte antigen (HLA-DQB1) gene variants and recurrent miscarriage.

**Methods:**

HLA-DQ gene polymorphisms (PCR-SSP) were detected in 50 couples with recurrent miscarriage (URSA group) and 30 couples with normal births (control group) using sequence-specific primer-guided polymerase chain reaction.

**Results:**

The frequency of the DQB1^*∗*^0303 allele in the URSA group (21.50%) was substantially higher than that of the control group (11.67%) (*P*=0.0260 0.05, RR = 1.754); however, the frequency of the DQB1^*∗*^0302 allele in the URSA group (4.00%) was substantially lower than that of the control pair (10.00%) (*P*=0.0318 0.05, RR = 0.400); the frequency of sharing one allele was 46.00% (23/50) in the URSA group and 0.00% (0/30) in the normal control group; the frequency of sharing two alleles was 40.00% (2/50) in the URSA group and 43.33% (13/30) in the normal control group, with no significant difference between the two groups.

**Conclusion:**

For the Zhejiang population, HLA-DQB1^*∗*^0303 may be a susceptibility gene for recurrent miscarriage, while HLA-DQB1^*∗*^0302 may be protective against recurrent miscarriage, especially for women.

## 1. Introduction

Recurrent spontaneous abortion (RSA) is a complex condition. Although it is defined nationally as 3 or more pregnancy losses, most experts believe that 2 spontaneous abortions should be taken seriously and evaluated because the likelihood of recurrent spontaneous abortion is similar to that of 3 [1]. RSA is defined by the American Society for Reproductive Medicine as two or more failed pregnancies occur within 20 weeks [2], with early miscarriages occurring before 12 weeks of gestation and late miscarriages occurring between 12 and 20 weeks of gestation [3], while the incidence of RSA in women of childbearing age is 3%–5% and the incidence of spontaneous abortion in repeat pregnancies in patients with RSA is as high as 70%–80% [4]. The etiology of RSA is complex and diverse, and in addition to genetic, anatomical abnormalities, endocrine disorders, infections, autoimmunity, sperm quality, lifestyle, psychosomatic, and environmental factors, the etiology of 50%–75% of RSA is still unknown [5]. The literature [6] shows that a significant proportion of recurrent spontaneous abortions are associated with immune factors. The HLA gene system is the most complex polymorphic system known in humans, and it has an important influence on the way the human immune system is regulated. The DQB1 allele polymorphism in the HLA-II class system is relatively high and has been shown to be significantly associated with recurrent abortions [7]. Considering the role of the HLA gene system in recurrent spontaneous abortion and its ethnic and geographical differences [8], the aim of this study was to investigate the role of the HLA gene system in recurrent spontaneous abortion by examining HLA-DQB1 gene polymorphisms in couples presenting with unexplained recurrent spontaneous abortion in Zhejiang province.

## 2. Material and Methods

### 2.1. Research Subjects

Fifty women who suffered from recurrent abortion were selected from October 2017 to February 2019 in Huzhou Central Hospital. All cases were selected after detailed history collection and auxiliary examination, and the following conditions were met at the same time: ① Two or more times of primary spontaneous abortion occurred continuously (2–10 times), and the last time occurred within 1 year; ② the bilateral chromosomes of the couple were normal; ③ the woman had no anatomical deformity of the reproductive tract, and abnormal internal secretion was excluded from the determination of the endocrine hormone level; ④ there was no infection in the reproductive system; ⑤ the results of autoimmune antibodies such as antiphospholipid antibodies were negative; ⑥ regular testing revealed that the male spouse's sperm was healthy. In the control group, 30 healthy expectant and postpartum women and their husbands who were hospitalized to the Obstetrics Department of Huzhou Central Hospital for delivery and underwent physical examination between November 2017 and March 2019 were chosen at random. There was no history of spontaneous abortion, stillbirth, coinfection, or autoimmune diseases in the control group. All the subjects were from Zhejiang province.

### 2.2. Research Methods

200 ul of EDTA anticoagulated whole blood was collected, and DNA was extracted using a DNA extraction kit at a concentration of 40–90 ng/uL and 1.7–2.0 at 260D/280D d. The HLA-DQB l locus was genotyped in strict accordance with the operating procedures of Tianjin Xiupeng Biotechnology Development Co., Ltd., and the results were interpreted by automatic analysis software. The review approach used PCR-SBT or sequence-based PCR typing.

### 2.3. Statistical Method

The frequencies of each allele were calculated by Microsoft Office Excel2003, with the analytic program SPSS17.0. The HLA-DQBl gene frequencies between the URSA group and the control group were compared using the chi-square test. The difference was statistically significant at *P* < 0.05. A relative risk calculation was made.

## 3. Result

### 3.1. Frequency Distribution of HLA-DQB1 Alleles

As shown in Table 1, the frequency of the HLA-DQB1^*∗*^0303 allele was 21.50% (43/200) in the URSA group and 11.67% (14/120) in the normal control group; the prevalence of the HLA-DQB1^*∗*^0303 allele was substantially higher in the URSA group than in the normal control group, *χ*^2^ = 4.954, *P*=0.026, and the frequency of the HLA-DQB1^*∗*^0302 frequency was 4.00% (8/200) in the URSA group and 10.00% (12/120) in the normal control group, *χ*^2^ = 4.608, *P*=0.032, histogram in Figure 1; as shown in Table 2, the HLA-DQB1^*∗*^0302 allele was significantly less frequent in the URSA female group with a frequency of 4.00% (4/100). The frequency was 13.33% (8/60) in the normal control female group, *χ*^2^ = 4.709, *P*=0.030, and there were no significant differences in the frequencies of other alleles (*P* > 0.05); the bar graphs are shown in Figure 2.

### 3.2. Sharing Rate of the HLA-DQB1 Allele between Couples

The frequency of sharing one allele was 46.00% (23/50) in the URSA couple group and 43.33% (13/30) in the normal control group, with no significant difference between these two groups, and the frequency of sharing two alleles was 40.00% (2/50) in the URSA couple group and 0.00% (0/30) in the normal control group.  Table 3 shows that there were no significant differences, and the bars are shown in Figure 3.

## 4. Discussion

### 4.1. Polymorphisms and Characteristics of the HLA-DQB1 Gene

Since the discovery of the first human leukocyte antigen Mac (HLA-A2) by French physician Dausset in 1958, research on HLA has developed rapidly [9]. HLA is located in region 21.3 of the short arm of chromosome 6, with a length of 4100 kb, and is by far the most polymorphic system known in humans, accounting for about 0.1% of the genes in the human genome [10]. The gene structure of this region has the following characteristics: (1) the region with the highest concentration and abundance of genes related to immune function, with 39.8% of gene products being immune among 128 functional genes; (2) the region with the highest gene density, with an average of one gene per 16 kb; (3) the region with the strongest polymorphism; (4) the region with the closest relationship to disease. In 1991, Bodmer classified HLA into three categories, namely, HLA-I genes including HLA-A, B, C, E, F, and G. HLA-II genes consist of six subunits, including HLA-DR, DQ, DP, DNA, DOB, and DM [11]. The HLA-III gene region mainly encodes complement-related genes, such as C2, C4A, C4B, and BF. In DQ of the HLA-II gene subregion, there are two pairs of *α* and *β* genes, of which, *α*1 and *β*1 domains are polymorphic sites and HLA-DQB1 is located in the *β*1 domain. A major function of the HLA-II gene is to present antigens and activate T lymphocytes, which are mostly present on the surface of dendritic cells, macrophages, B lymphocytes, activated T lymphocytes, and other cells. The distribution of HLA is ethnic and regional, and the genetic characteristics of HLA gene frequencies vary among different ethnic and regional populations [12].

### 4.2. HLA Gene System and Immunity

The HLA gene system has a major impact on the way the human immune system is regulated. The literature [13] showed that whether the body responds to antigenic substances and the intensity of the response is genetically controlled. The HLA class II gene region contains immune response regulatory genes. Due to the different peptide structures of the molecules encoded by HLA-II genes, their ability to bind different antigenic peptides and stimulate Th cells is different, so the expression of genes in the immune response is different. The non-T cell surface stimulation of autologous mixed lymphocytes in response to AMLR is determined by HLA-DQ in one of the HLA-II molecules. AMLR is a regulatory mechanism between immune cells in vivo, maintaining immune homeostasis. Thus, by activating AMLR, HLA-II-like molecules can influence immunological control. Despite the fact that the fetus is a semiallogeneic transplant of the mother, the immune response of the mother during pregnancy can protect the fetus from rejection. However, the literature [14] has demonstrated that several tolerance mechanisms limit the maternal immune response during normal pregnancy. The literature [15] showed that in couples with unexplained recurrent spontaneous abortions, HLA molecules are thought to have played an important role at the maternal-fetal interface. Fetal blood enters the maternal circulation when exchanging blood with the mother through the placenta, and the maternal immune system is able to recognize paternal HLA antigens carried by the blood; excessive sharing of HLA antigens between the couple can lead to insufficient production of blocking antibodies and finally to recurrent miscarriage. The literature [16] suggests that excessive sharing of HLA antigens between couples can lead to low maternal responsiveness to paternal antigens, which is an important mechanism leading to recurrent miscarriage. The literature [17] suggests that antipaternal HLA antibodies may not be harmful in healthy pregnancies but rather may even be beneficial. However, the literature [18] suggests that maternal HLA antibodies are detrimental to pregnancy in couples with recurrent miscarriage.

### 4.3. Undiagnosed Recurrent Miscarriage and HLA-DQB1 Gene Polymorphism

In this study, 50 couples with URSA and 30 couples with normal births were studied. The results showed that HLA-DQB1^*∗*^0303 may be a susceptibility gene for recurrent miscarriage and that HLA-DQB1^*∗*^0302 may play a protective role against recurrent miscarriage, especially in women. Studies in the literature [19] suggest that DQB1^*∗*^03 : 03 : 02 is a susceptibility gene for recurrent miscarriage in South India, and the inconsistent results may be due to regional and ethnic differences in HLA. A study in the literature [20] showed that the number of couples sharing two HLA alleles for recurrent pregnancy loss was less than those sharing one allele and those not sharing, and the rate of HLA allele sharing did not correlate with recurrent miscarriage. The results of this study showed that there was no significant difference in the frequency of sharing one allele between URSA couples and normal controls, nor was there a significant difference in the frequency of sharing two alleles between URSA couples and normal controls. The results of this study also show a lack of association between the rate of HLA allele sharing and unexplained recurrent miscarriage. In addition, it needs to be compared with epidemiological data on the population distribution of HLA-DQB1 in China. The literature [18] on the distribution of HLA-DQB1 polymorphisms in South and North China showed that the distribution of HLA-DQB1^*∗*^02, 05, 0601, 0602, and 0603 in the Chinese population was different between North and South. The literature [21] reported that HLA-DQB1^*∗*^0303, 0302 did not differ significantly between North and South China. However, few studies have examined the distribution of HLA-DQB1 allele polymorphisms in Zhejiang. Due to the vast geographical area and many ethnic groups in China, the sample data of HLA-DQB1 in unexplained recurrent miscarriage need to be expanded and epidemiological data need to be improved.

## Figures and Tables

**Figure 1:** Frequency distribution of HLA-DQB1 alleles in 50 URSA couples and 30 normal fertile couples.

**Figure 2:** Frequency distributions of HLA-DQB1 alleles in 50 URSA females and 30 fertile females.

**Figure 3:** Comparison of the number of shared HLA-DQB1 alleles between 50 URSA couples and 30 fertile couples.

**Table 1:** Frequency distribution of HLA-DQB1 alleles in 50 URSA couples and 30 normal fertile couples.

HLA-DQB1 genotypes	Couples in the URSA group (*n* = 200)		Couples in the normal group (*n* = 120)		*χ* ^2^ value	*P* value
	Times	Frequency (%)	Times	Frequency (%)		
0301	49	24.50	31	25.83	0.0711	0.7897
0303	43	21.50	14	11.67	4.9541	0.026
0201	17	8.50	16	13.33	1.9671	0.1607
0501	18	9.00	14	11.67	0.5926	0.4414
0302	8	4.00	12	10.00	4.6081	0.0318
0202	10	5.00	5	4.17	0.1166	0.7328
0602	10	5.00	11	9.17	2.1231	0.1451
0401	10	5.00	6	5.00	0	1
0603	7	3.50	6	5.00	0.3169	0.5735
0503	6	3.00	3	2.50	0.0686	0.7934
0402	1	0.50	1	1.83	0.1342	0.7141
Total genotype	179		119			

**Table 2:** Frequency distributions of HLA-DQB1 alleles in 50 URSA females and 30 fertile females.

HLA-DQB1 genotypes	Females in the URSA group (*n* = 100)		Females in the normal group (*n* = 60)		*χ* ^2^ value	*P* value
	Times	Frequency (%)	Times	Frequency (%)		
0301	25	25.00	15	25.00	0	1
0303	21	21.00	7	11.67	2.2631	0.1325
0201	11	11.00	8	13.33	0.1951	0.6587
0501	10	10.00	6	10.00	0	1
0602	7	7.00	5	8.33	0.0961	0.7566
0401	5	5.00	3	5.00	0	1
0302	4	4.00	8	13.33	4.7091	0.03
0603	4	4.00	5	8.33	1.3261	0,2494
0402	1	1.00	1	1.67	0.135	0.7133
0202	2	2.00	1	1.67	0.2265	0.8804
Total genotype	90		59			

**Table 3:** Comparison of the number of shared HLA-DQB1 alleles between 50 URSA couples and 30 fertile couples.

Allelic genes	URSA group (*n* = 50)		Normal group (*n* = 30)		*χ* ^2^ value	*P* value
	Times	Frequency (%)	Times	Frequency (%)		
Share 1 allelic gene	23	46.00	13	43.33	0.0539	0.8165
Share 2 allelic genes	2	4.00	0	0.00	1.2311	0.2673

## Data Availability

The data used to support the findings of this study are available from the corresponding author upon request.
